RETRACTED

# Effects of DNA Immunoadsorption Combined with Medication on Immune Function and Renal Function in Patients with Systemic Lupus Erythematosus

**DOI:** 10.1155/2023/2843979

**Published:** 2023-02-21

**Authors:** Lijie Bai, Mingxia Sun, Guiying Wu, Jing Wang, Yong Wang, Jun Shi, Liying Zhang

**Affiliations:** ^1^Department of Rheumatology, Affiliated Hospital of Inner Mongolia Medical University, Huhehaote 010059, China; ^2^Department of Nephrology and Rheumatology, Hohhot First Hospital, Huhehaote 010000, China; ^3^Inner Mongolia Medical University, Huhehaote 010059, China; ^4^Department of Nephrology, Affiliated Hospital of Inner Mongolia Medical University, Huhehaote 010059, China

## Abstract

*Objective*. At present, glucocorticoids combined with cyclophosphamide are still used for the clinical treatment of systemic lupus erythematosus (SLE). However, long-term practice has shown that drug treatment currently has the phenomena of long treatment duration, uncontrollable conditions in a short period of time, and unsatisfactory efficacy. DNA immunoadsorption therapy is a newly developed therapy. The combination of drugs and DNA immunoadsorption has been reported for the treatment of SLEN in clinics for a long time. In this study, we observed the effects of DNA immunoadsorption combined with drug therapy on immune function and renal function in patients with systemic lupus erythematosus (SLE). The results showed that the DNA immunosorbent assay combined with medication in the treatment of SLE could quickly and specifically remove pathogenic substances from patients, improve renal function, immune function, and complement levels in patients, and help to relieve disease activity.

## 1. Introduction

Systemic lupus erythematosus (SLE) is an autoimmune, inflammatory connective tissue disease involving multiple organs that occurs mostly in young women. Its clinical manifestations are complex and varied, which can lead to changes in brain, kidney, blood, skin, and joints [1]. Immunosuppressive agents are mainly used in clinics to inhibit abnormal immune and inflammatory responses in order to treat SLE [2]. In recent years, with the continuous improvement of treatment methods, the use of hormones and immunosuppressants, and the emergence of biological agents, the prognosis of SLE patients has greatly improved. However, immunosuppressive agents have poor efficacy for patients with high activity of SLE, especially for patients with combined nervous system lesions. Moreover, such patients have become the difficulties in the treatment of SLE due to their rapid disease progression, poor treatment response, and poor clinical prognosis [3]. At present, the early removal of autoantibodies from patients' serum, control of disease activity, and protection of renal function are the keys to treatment.

RETRACTED

DNA immunoadsorption is a new therapeutic method developed on the basis of plasma exchange. DNA is fixed on the carrier as a ligand to form an adsorption column, which can specifically remove the anti-DNA antibody or immunoglobulin by the biological affinity of antigen and antibody, thereby reducing the damage of pathogenic antibodies and immune complexes to tissues and organs [4]. A single treatment with a DNA immunosorbent assay can effectively eliminate endogenous pathogenic factors in blood of SLE patients, help patients survive an immune storm, and promote disease remission. Stummvoll et al. [5] observed that 16 patients with SLE nephritis had significantly improved resistance after three months of immunoadsorption treatment, with the SLE disease activity index (SLEDAI) score decreased, proteinuria significantly reduced, and anti-ds-DNA antibody titer decreased. These results indicated that the DNA immunosorbent assay could effectively control the condition of SLE patients and create the conditions for later drug treatment. In order to further verify this result, in this study, we investigated the effects of DNA immunoadsorption combined with glucocorticoids, cyclophosphamide, and other drugs on the immune function and renal function in patients with SLE in order to provide more evidence for the clinical treatment of SLE.

## 2. Data and Methods

### 2.1. General Information

A total of 84 patients with SLE who visited our hospital from May 2018 to May 2021 were selected. According to the difference in treatment methods, all patients were divided into an observation group and a control group, with 42 cases in each group.

### 2.2. Inclusion and Exclusion Criteria

#### 2.2.1. Inclusion Criteria

The inclusion criteria were as follows: all patients met the diagnostic criteria for SLE, no treatment with glucocorticoids or immunosuppressive drugs within 2 months before treatment, patients with 24 h urine protein quantification in the urine test ≥1 g, and patients with normal coagulation function and no bleeding tendency or active bleeding.

#### 2.2.2. Exclusion Criteria

The exclusion criteria were as follows: patients with combined renal malignant tumor, patients with severe cardiovascular and cerebrovascular diseases, patients with severe bacterial or active viral infections such as hepatitis B and C, patients with a history of acute rheumatic fever and rheumatoid arthritis, patients who are allergic to the drugs used in this study, and women who are pregnant or nursing.

### 2.3. Treatment Methods

Patients in the control group were treated with the conventional medication for SLE, namely, glucocorticoids combined with cyclophosphamide pulse therapy. Methylprednisolone tablets were administered at a dose of 0.8 mg/(kg·d) once per day. Cyclophosphamide (0.5 g) for injection was added into 250 mL of 0.9% sodium chloride solution for intravenous infusion once every 2 weeks and changed to once every 4 weeks after 6 weeks according to the degree of disease of the patient. Continuous treatment was given for 6 months.

RETRACTED

On the basis of the control group, patients in the observation group were treated with DNA immunoadsorption. A DNA immunoadsorption column, a hemoperfusion machine, and extracorporeal circulation equipment were used for the adsorption treatment. Specific steps were as follows: 500 mL of 5% glucose injection was added into the adsorption column and allowed to stand for 30 min. During the static period, gently tap and rotate the adsorption column every 10 minutes for 1 to 2 minutes. After the adsorbent particles are saturated, use 4000 mL of heparin sodium and sodium chloride solution to flow in the adsorption system of the adsorption column from top to bottom, with a flow rate of 50 to 100 mL/min. Gently tap and rotate the adsorption column with your hand until the exhaust is exhausted. Finally, use 500 mL of heparin sodium chloride solution (including 100 mg of heparin) to close the circulation for 30 minutes to make the adsorption column completely heparinized. After successful deep venipuncture of bilateral iliac venous access, intravenous heparin was started at a dose of 1 mg/kg body weight with a total dose of 16–20 mg/h, and heparin was stopped 30 min before the end. After the deep vein indwelling catheter was effectively connected to the adsorption column as the vascular access, a preflush was performed and connected to the venous line so that the patient could establish effective cardiopulmonary bypass and anticoagulation. The blood pump was started at an initial speed of 80–100 mL/min and then gradually increased to 100–150 mL/min. After adsorption, blood was returned using the air-to-blood method, and protamine was slowly injected intravenously to neutralize the heparin. The single adsorption time was 2-3 h, and the next treatment could be carried out after an interval of 3 d. According to the patient's tolerance and serological indicators, DNA immunoadsorption therapy was performed two to three times.

### 2.4. Observation Indicators

1. Health status evaluation: before and after treatment, clinical analysis was performed on 24 indicators of nine organ systems in patients according to the SLEDAI, with a total score of 105 points [6]. The basic inactive period is 0–4 points, the mild active period is 5–9 points, the moderate active period is 10–14 points, and the severe active period is ≥15 points. Meanwhile, using the MOSF-36 scale as a measurement tool and an anonymous survey, the physical function (PF) and mental health (MH) scores of the two groups before and after treatment were compared.
2. Detection of immune function: before and after treatment, 3 mL of fasting venous blood was collected from the patients. After centrifugation, the levels of immunoglobulins (IgA, IgG, and IgM), complement C3 and C4 were detected by electrochemical luminescence assay.
3. Detection of inflammatory factor indicators: before and after treatment, 3 mL of venous fasting blood was collected and centrifuged. Serum levels of interleukin-6 (IL-6), interleukin-8 (IL-8), and tumor necrosis factor-*α* (TNF-*α*) were measured by enzyme-linked immunosorbent assay.
4. Renal function test: before and after treatment, the peripheral blood of patients was collected, and after centrifugation, the blood urea nitrogen (BUN) and serum creatinine (SCr) contents were measured by the electrochemical luminescence method. The 24 h urine samples of patients were collected before and after treatment, and the urine protein content was detected by an automatic urine analyzer.
5. Adverse reactions: during the treatment, mild rash, thrombocytopenia, fever, malignant vomiting, and decreased blood pressure in the two groups were recorded.

RETRACTED

### 2.5. Statistical Methods

SPSS 22.0 software was used for processing. The measurement data that conformed to the normal distribution of the experimental data were expressed as mean ± SD. An independent sample *t*-test was used for comparison between groups. A paired *t*-test was used for intragroup comparison. Experimental data were counted and expressed as (%) and compared by the *x*^2^ test. The test level was *α* = 0.05, and *P* < 0.05 indicated that the difference was statistically significant.

## 3. Results

### 3.1. General Baseline

There was no significant difference in general baseline data between the two groups (*P* > 0.05), as shown in Table 1.

### 3.2. Assessment of the Health Status of Patients in Two Groups

Before treatment, the SLEDAI score, PF score, and MH score between the two groups were not statistically significant (*P* > 0.05). After treatment, the SLEDAI score of patients in the observation group was lower than that of the control group, and the PF score and MH score of patients in the observation group were higher than those of patients in the control group (both *P* < 0.05), as shown in Figure 1.

### 3.3. Comparison of Immune Indexes between the Two Groups

Before treatment, the levels of IgA, IgG, IgM and complement C3 and C4 between the two groups were not statistically significant (*P* > 0.05). After treatment, the levels of IgA, IgG, and IgM in patients of the observation group were lower than those of the control group, and the levels of complement C3 and C4 were higher than those of the control group (all *P* < 0.05), as shown in Table 2.

RETRACTED

### 3.4. Comparison of Inflammatory Factor Levels between the Two Groups

Before treatment, the levels of IL-6, IL-8, and TNF-*α* between the two groups were not statistically significant (*P* > 0.05). The levels of IL-6, IL-8, and TNF-*α* in the two groups of patients after treatment were lower than those before treatment, and the levels of IL-6, IL-8, and TNF-*α* in the observation group were lower than those in the control group (all *P* < 0.05), as shown in Figure 2.

### 3.5. Comparison of Renal Function Indexes between the Two Groups

Before treatment, the levels of BUN and SCr and the 24 h urinary protein quantity between the two groups were not statistically significant (*P* > 0.05). The levels of BUN and SCr and 24 h urinary protein quantity in the two groups after treatment were lower than those before treatment, and the levels of BUN and SCr and 24 h urinary protein quantity in the observation group were lower than those in the control group (all *P* < 0.05), as shown in Figure 3.

### 3.6. Adverse Reactions in Two Groups during Treatment

In the observation group, there were three cases of mild rash, one case of thrombocytopenia, three cases of generate heat, four cases of nausea and vomiting, and one case of decreased blood pressure, with the total incidence rate of 28.57%. In the control group, there were two cases of mild rash, two cases of generating heat, and three cases of nausea and vomiting, with a total incidence rate of 16.67%. There was no statistical significance in the incidence rate of various adverse reactions or the total incidence between the two groups (all *P* > 0.05), as shown in Table 3.

## 4. Discussion

At present, the principle of clinical treatment of SLE is “classification, staging, combination, and long-term,” and the drugs used target control immunosuppressants and cytotoxic drugs with the ultimate goal to inhibit excessive autoimmune responses [7, 8]. Autoantibodies in SLE patients can attack their cells and tissues, forming antigen-antibody complexes that are deposited in the vascular wall, glomerular basement membrane, and other areas, eventually leading to target organ function damage [9, 10]. Glucocorticoids combined with cyclophosphamide have anti-inflammatory and anti-T-lymphocyte proliferation effects, which can alleviate the clinical symptoms of patients [11, 12]. However, in the process of conventional drug treatment, it will inhibit the body's immune function and the resulting cytotoxicity, resulting in a poor anti-inflammatory effect. In recent years, biological agents for the treatment of SLE have appeared, but most of them are still in the initial stages of research and clinical application, and their efficacy and safety await follow-up and evaluation in large-scale double-blind controlled trials.

RETRACTED

The results of this study showed that the improvement in SLEDAI, PF, and MH scores was better in the treatment group than in the control group. SLEDAI is recognized as a reliable and effective tool for evaluating the activity of SLE [13]. Therefore, this result indicates that the clinical application of immunoadsorption, hormones, and immunosuppressants can effectively remove antibodies from the body and alleviate the symptoms of patients with exact clinical efficacy. DNA immunoadsorption therapy is an emerging method for the treatment of autoimmune diseases in recent years, which belongs to the field of blood purification treatment [14, 15]. DNA immunoadsorption therapy uses antigens or other substances with specific physicochemical affinity as ligands, which are combined with the carrier and connected to the adsorption column. Specific adsorption is used to eliminate endogenous pathogenic factors in patients' blood, so as to exert the effects of purifying blood, eliminating immune complexes and immunoglobulins in patients with SLE, alleviating target organ damage, and achieving the effects of targeted therapy for SLE [16, 17].

Studies have found that the body's immune function, complement, and inflammatory factor levels are closely related to the occurrence and development of SLE [18]. The insufficient production of inhibitory T lymphocytes will result in the weakened inhibition of CD8+ T cells on B lymphocytes, which in turn leads to the abnormal proliferation of B lymphocytes and the secretion of a large amount of Ig, thereby increasing the content of Ig in the body and accelerating the further development of the patient's condition [19]. In addition, complement is also involved in the regulation of immune function and the formation of antigen-antibody complexes. Complement C3 and C4 are glycoproteins with enzyme activity in body fluids. There are a large number of autoantibodies in SLE patients, and their phagocytosis in the formed antigen-antibody complex will consume a large amount of complement, resulting in a reduction of complement content in the body [20, 21]. In this study, DNA immunoadsorption combined with medication significantly reduced IgA, IgG, and IgM levels in patients and increased complement C3 and C4 levels in patients. It indicated that DNA immunoadsorption therapy combined with medication could improve the high immune function of patients. The reason for this is that DNA immunoadsorption therapy could eliminate autoantibodies in vivo in time, so as to regulate immune function and restore balance.

RETRACTED

The results of this study showed that the levels of inflammatory factors were decreased after treatment in both groups compared with those before treatment, and they were significantly better in the observation group than in the control group patients. IL-6 can stimulate the activation and differentiation of inflammatory cells, aggravating the inflammatory damage to the target organs in SLE patients and the progression of the disease. The massive release of IL-8 in the active stage of SLE disease further aggravates the renal inflammatory response [22, 23]. TNF-*α* is a widely used cytokine in clinics; its level can be significantly elevated when the body is stimulated by external bacteria and viruses. The significant difference in IL-6, IL-8 and TNF-*α* after treatment between the two groups in this study may be due to the fact that DNA immunosorbent assay could remove endogenous pathogenic factors such as autoantibodies and inflammatory factors in blood through specific adsorption and reduce complement consumption in patients' bodies, which plays a role in improving immune function of patients, increasing complement level, and reducing inflammatory factor level in vivo.

SLE can involve multiple organs throughout the body, with kidney involvement being the most severe. When the kidneys are involved, SLE patients will present with such symptoms as hematuria, proteinuria, and edema or even lead to end-stage renal disease, which will endanger the patients' lives [24, 25]. The local deposition of antigen-antibody complexes in the glomeruli is the most fundamental pathological change leading to renal impairment [26, 27]. Braun et al. [28] adopted immunoadsorption to treat SLE patients with routine immunosuppressive resistance, and 70% of the patients recovered within three weeks after treatment with rapid reduction of circulating immune complexes and immunoglobulins, serum SCr reduction, and significantly reduced urine protein. DNA immunoadsorption therapy can directly remove autoantibodies, especially anti-ds-DNA antibodies, which are closely related to the prognosis, so as to reduce the damage of the antigen-antibody complex to the glomerulus [29, 30]. Therefore, the results of this study show that the BUN and SCr levels and 24 h urine protein quantity in the observation group were lower than those in the control group. This further confirms that DNA immunosuppression combined with glucocorticoid and cyclophosphamide treatment might help to improve the renal function in patients with SLE.

RETRACTED

Our study further observed the occurrence of adverse reactions in the two groups and found that the combination of DNA immunosuppression and drug treatment did not increase the adverse reactions of the patients, which is beneficial for the patients to safely survive the highly active clinical risk period of the condition. It should also be noted that although the use of glucocorticoids and immunosuppressive agents during treatment can significantly improve the clinical outcome and prognosis of patients, the 5-year survival rate of approximately 10% of patients is still poor. Therefore, once clinically diagnosed, effective treatment measures that inhibit lupus activity are taken immediately to ensure the improvement of clinical symptoms and further improve the prognosis. At the same time, shortening the medication time as much as possible during the induction treatment stage is also the key to ensure the long-term prognosis of patients and reduce complications [31].

To sum up, a DNA immunosorbent assay combined with drugs in the treatment of SLE can quickly and specifically remove pathogenic substances from patients, improve renal function, immune function, and complement levels in patients, and help to relieve disease activity. However, its exact effect and long-term efficacy require further evidence from large samples and multicenter prospective trials.

## Figures and Tables

**Figure 1:** Health status evaluation of two groups of patients. (a) SLEDAI score. (b) PF score. (c) MH score. (^*∗*^*P* < 0.05).

**Figure 2:** Comparison of inflammatory factor levels between the two groups. (a) IL-6. (b) IL-8. (c) TNF-*α*. (^*∗*^*P* < 0.05).

**Figure 3:** Comparison of renal function indicators between the two groups. (a) BUN. (b) SCr. (c) 24 h urine protein quantification. (^*∗*^*P* < 0.05).

**Table 1:** Comparison of general baseline information between the two groups.

	Control group (*n* = 42)	Observation group (*n* = 42)	*x* ^2^ * /t*	*P*
Gender (*n* (%))			0.060	0.806
Male	11	12		
Woman	30	29		
Mean age (years, *x* ± *s*)	33.95 ± 4.29	34.16 ± 4.07	0.230	0.819
Mean course of disease (years, *x* ± *s*)	2.16 ± 0.67	2.14 ± 0.64	0.140	0.889
SLEDAI score (score, *x* ± *s*)	22.07 ± 0.94	21.92 ± 0.87	0.759	0.450
Organ involvement (*n* (%))			0.135	0.987
Central nervous system	29	30		
Heart	27	28		
Lungs	21	19		
Kidney	41	41		
White blood cells (×10^9^/L, *x* ± *s*)	5.35 ± 1.14	5.28 ± 1.37	0.255	0.799
Hemoglobin (g/l, *x* ± *s*)	96.84 ± 12.53	95.71 ± 10.96	0.051	0.960
Platelets (×10^9^/L, *x* ± *s*)	216.74 ± 41.27	224.89 ± 42.73	0.889	0.377

RETRACTED

**Table 2:** Comparison of immune indexes between the two groups.

Group	Time	IgA (g/L)	IgG (g/L)	IgM (g/L)	C3 (g/L)	C4 (g/L)
Control group (*n* = 42)	Before treatment	2.63 ± 0.41	20.95 ± 3.38	1.84 ± 0.42	0.51 ± 0.07	0.07 ± 0.02
	After treatment	2.54 ± 0.38^a^	18.52 ± 3.12^a^	1.72 ± 0.33^a^	0.54 ± 0.02^a^	0.08 ± 0.01^a^

Observation group (*n* = 42)	Before treatment	2.61 ± 0.43	20.49 ± 3.26	1.86 ± 0.45	0.50 ± 0.06	0.07 ± 0.01
	After treatment	2.42 ± 0.29^ab^	16.37 ± 2.81^ab^	1.63 ± 0.30^ab^	0.57 ± 0.05^ab^	0.09 ± 0.03^ab^

**Table 3:** Comparison of adverse reactions between the two groups.

Group	Mild rash	Thrombocytopenia	Generate heat	Nausea and vomiting	Decreased blood pressure	Total incidence
Control group (*n* = 42)	2 (4.76)	0 (0.00)	2 (4.76)	3 (7.14)	0 (0.00)	7 (16.67)
Observation group (*n* = 42)	3 (7.14)	1 (2.38)	3 (7.14)	4 (9.52)	1 (2.38)	12 (28.57)
*x* ^2^	0.213	1.012	0.213	0.156	1.012	1.700
*P*	0.645	0.314	0.645	0.693	0.314	0.192

## Data Availability

The data used to support the findings of this study are available from the corresponding authors upon request.
